# Hyperbaric oxygen therapy as rescue therapy for pediatric frosted branch angiitis with Purtscher-like retinopathy: A case report

**DOI:** 10.3389/fmed.2023.1119623

**Published:** 2023-04-17

**Authors:** Chi-Tai Lee, Tzu-Han Hsieh, Chan-Ching Chu, Yung-Ray Hsu, Jia-Horng Wang, Jia-Kang Wang, Zhanqi Zhao, Hou-Tai Chang

**Affiliations:** ^1^Center of Hyperbaric Oxygen, Far Eastern Memorial Hospital, New Taipei City, Taiwan; ^2^Department of Chest Medicine, Far Eastern Memorial Hospital, New Taipei City, Taiwan; ^3^Department of Ophthalmology, Far Eastern Memorial Hospital, New Taipei City, Taiwan; ^4^Department of Electrical Engineering, Yuan Ze University, Taoyuan, Taiwan; ^5^Department of Critical Care Medicine, Far Eastern Memorial Hospital, New Taipei City, Taiwan; ^6^Department of Biomedical Engineering, Fourth Military Medical University, Xi’an, China; ^7^Institute of Technical Medicine, Furtwangen University, Villingen-Schwenningen, Germany; ^8^Department of Industrial Engineering and Management, Yuan Ze University, Taoyuan, Taiwan

**Keywords:** frosted branch angiitis, Purtscher-like retinopathy, hyperbaric oxygen therapy, positive antinuclear antibody, atmosphere absolute, best-corrected visual acuity, optical coherence tomography

## Abstract

**Introduction:**

Frosted branch angiitis (FBA) is an uncommon uveitis characterized by fulminant retinal vasculitis. Purtscher-like retinopathy (PuR) is a rare retinal angiopathy associated with a non-traumatic etiology. Both FBA and PuR can cause profound visual impairments.

**Case report:**

We describe the case of a 10-year-old male who presented with sudden bilateral painless visual loss due to FBA with concurrent PuR, with notable viral prodrome 1 month prior to presentation. Systemic investigations revealed a recent herpes simplex virus 2 infection with a high titer of IgM, positive antinuclear antibody (ANA) (1:640), and abnormal liver function tests. After administration of systemic corticosteroids, anti-viral agents, and subsequent immunosuppressive medications, the FBA was gradually alleviated. However, fundoscopy and optical coherence tomography (OCT) revealed persistent PuR and macular ischemia. Hence, hyperbaric oxygen therapy was administered as a rescue strategy, which resulted in gradual bilateral visual acuity improvement.

**Conclusion:**

Hyperbaric oxygen therapy may be a beneficial rescue treatment for retinal ischemia secondary to FBA with PuR.

## Introduction

Uveitis is a group of ocular inflammatory diseases encompassing non-infectious and infectious causes. Frosted branch angiitis (FBA) is an uncommon retinal vasculitis characterized by widespread perivascular sheathing that simulates frost on a tree branch. Apart from lymphoma or leukemic cell infiltration, or definite infectious diseases such as cytomegalovirus retinitis, most reported cases of FBA are idiopathic, with presumed viral prodromes before the ocular manifestations (1).

Purtscher-like retinopathy (PuR) is a clinical phenomenon characterized by diffuse white plaques, namely Purtscher fleckens confined within the macular area, with precapillary arteriole occlusion. Optical coherence tomography (OCT) often reveals the pattern of paracentral acute middle maculopathy (2). PuR results from various non-traumatic etiologies (3), and among which, viral infections are extremely rare.

Hyperbaric oxygen therapy (HBOT) has been used to treat blindness, including central retinal artery occlusion, macular edema due to diabetes, and specific optic neuropathy (4–6). We report a case utilizing HBOT as a rescue treatment for macular ischemia in post-viral infection-induced FBA and PuR.

## Case report

A 10-year-old male consulted our ophthalmology department due to bilateral blurred vision for one week. He had experienced a 1-week episode of flu-like symptoms, including fever and general malaise, 1 month before the ocular presentation. The best-corrected visual acuity (BCVA) was 0.025 (both eyes, BE). The intraocular pressure was within the normal range. Slit lamp examinations revealed 0.5+ anterior chamber cells (BE) with otherwise normal anterior segment structures. Indirect ophthalmoscopy revealed bilateral diffuse perivascular sheathing of the arteries and veins, Purtscher fleckens, and mild optic papillitis. Necrotizing retinitis was not observed (Figures 1A, B). OCT revealed profound macular edema with intraretinal fluid, subretinal fluid, and inner to middle retinal layer hyperreflectiveness (Figure 2A). Ultrawide-field fluorescein angiography revealed bilateral segmental phlebitis, occlusive arteritis, and retinal non-perfusion with macular ischemia. Due to previous systemic prodromes, a pediatrician was consulted for multidisciplinary care.

**FIGURE 1:** Serial ultrawide-field fundus photographs. **(A)** Initial presentation showed diffuse perivascular sheathing with frosted branch angiitis appearance. **(B)** Initial fluorescein angiography revealed multiple segmental phlebitis (yellow arrow) with occlusive arteritis (white arrow) and retinal non-perfusion (orange arrow). The visual acuity was 0.025 (both eyes). **(C)** Four weeks later, partial resolution of the perivasculitis following systemic corticosteroid and antiviral treatment was seen; however, aggravated Purtscher-like retinopathy was demonstrated (white arrow). **(D)** Twenty-one weeks after initial visit and 8 weeks following HBOT, alleviated vascular leakage, however, with extensive macular and midperipheral retinal non-perfusion was shown. The visual acuity was 0.16 (both eyes). **(E)** Nineteen weeks after initial visit, reduced Purtscher fleckens was note. Frosted branch angiitis almost completely resolved following combined corticosteroid, antiviral agent, and immunosuppressive medications. **(F)** Thirty-nine weeks after initial visit and 26 weeks following HBOT as well as 15 weeks after retinal photocoagulation, there were vascular leakage with few vitreous hemorrhage. The visual acuity was 0.1 (right) and 0.16 (left).

**FIGURE 2:** Serial changes in OCT. **(A)** Initial OCT showed profound macular edema with combine intraretinal and subretinal fluid. **(B)** Two weeks after initial visit, partial resolution of the macular edema; however, hyperreflective change could be noted at the inner and middle retinal layers. The visual acuity was 0.1 (right) and 0.05 (left). **(C)** Eleven weeks after initial visit, complete resolution of the macular edema. CFT 156 μm (right) and 147 μm (left). The visual acuity was 0.05 (right) and counting finger 30 cm (left). **(D)** Seventeen weeks after initial visit and 4 weeks following HBOT. Slightly reduce hyperreflectivity at the left eye could be noted. The visual acuity was 0.1 (both). **(E)** Twenty-one weeks after initial visit and 8 weeks following HBOT. Extensive retinal thinning with ellipsoid zone loss was noted. The visual acuity was 0.16 (both). **(F)** Twenty-eight weeks after initial visit and 15 weeks following HBOT. Reduced inner retinal thinning was noted. The visual acuity was 0.16 (right) and 0.2 (left). **(G)** Forty-three weeks after initial visit and 30 weeks following HBOT. Reduced inner retinal thinning was noted. The visual acuity was 0.05 (right) and 0.16 (left). **(H)** Sixty weeks after initial visit and 47 weeks following HBOT. Reduced inner retinal thinning was noted. The visual acuity was 0.1 (right) and 0.16 (left).

Physical examination results aside from the ocular findings were unremarkable. Abdominal ultrasonography revealed mild hepatomegaly. Initial hematology and serology investigations revealed an elevated erythrocyte sedimentation rate at 58 mm/h, alanine aminotransferase at 160 U/L, and positive antinuclear antibody (1:640). A systemic infection survey targeting retinal vasculitis and hepatitis revealed negative results for HSV-1, CMV, VZV, EBV, HTLV, HBV, HCV, Quantiferon-TB Gold, syphilis, and toxoplasma serology. However, a highly positive titer of HSV 2 IgM (5.10) was noted. An aqueous tap was not performed because of its invasiveness considering the age of the patient. In addition, the associated autoimmune profiles were positive for anti-smooth muscle antibody (Ab), but negative for anti-dsDNA, anti-mitochondria Ab, or anti-liver kidney microsome Ab (anti-LKM Ab). Therefore, this patient was diagnosed with post-HSV-2 infection-related FBA, PuR, and concurrent autoimmune hepatitis. The patient was initially prescribed prednisolone (40 mg/day), valaciclovir (500 mg every 12 h), and acetylsalicylic acid (100 mg every other day) (Figure 3).

**FIGURE 3:** Treatment timeline. ATA, atmosphere absolute; HBOT, hyperbaric oxygen therapy; qd, every day; q12h, every 12 hours; qod, every other day; qw, every week. *Treatment protocol: 2.0 ATA for 75 min per session, 1 session per day, 5 days per week.

Although the bilateral FBA and macular edema gradually alleviated (Figures 1C, 2B) after several weeks of medical treatment, the BCVA improvement was minimal (0.05, right eye; counting finger, left eye) (Table 1). Persistent macular ischemia, with clinical presentations of profound PuR and compatible ischemic hyperreflective changes on OCT (Figures 1C, 2C), was identified to be the main cause of poor vision. Therefore, HBOT was initiated with 2.0 atmosphere absolute (ATA) for 75 min per session, 1 session per day, 5 days per week. After a total of 39 sessions of HBOT, the visual acuity steadily improved to 0.16 (RE) and 0.2 (LE), with gradual resolution of Purtscher fleckens (Table 1). Subsequent immunosuppressive medications, including methotrexate (10 mg/week) and cyclosporine (50 mg/day), were also initiated for FBA treatment and corticosteroid tapering (Figure 3). Follow-up fundus photograph and fluorescein angiography performed 21 weeks after the initial visit and 8 weeks following HBOT revealed almost completely resolution of FBA and decrease in size of PuR, but extensive macular and mid-peripheral retinal ischemia (Figures 1D, E). Therefore, retinal photocoagulation on the non-perfusion area was performed 13 weeks after the initiation of HBOT to prevent further neovascular complications, such as vitreous hemorrhage, tractional retinal detachment, and neovascular glaucoma (Figure 1F).

**TABLE 1:** Hyperbaric oxygen therapy sessions and visual acuity and ocular findings monitoring.

Week	HBOT (cumulative sessions)*	BCVA		CFT (μm)	
		**OD**	**OS**	**OD**	**OS**
Initial	0	0.025	0.025	394	396
2nd week	0	0.1	0.05	320	210
5th week	0	0.1	0.16	204	196
11th week	0	0.05	CF 30 cm	156	147
15th week	12	0.1	CF 20 cm	153	137
17th week	22	0.1	0.1	152	142
19th week	30	0.1	0.1	155	140
21st week	30	0.16	0.16		
28th week	39	0.16	0.2	158	143

HBOT, hyperbaric oxygen therapy; BCVA, best-corrected visual acuity; CFT, central foveal thickness on optical coherence tomography; OD, right eye; OS, left eye.

*Treatment protocol: 2.0 atmosphere absolute (ATA) for 75 min per session.

## Discussion

This case raises three important issues for clinicians. First, the clinical appearance of the fundus showed typical FBA; however, the clinical course was prolonged compared to typical FBA cases. Second, with bilateral retinal vasculitis and high titer of HSV-2 IgM in the serology survey, non-necrotizing herpetic retinopathy, which is the immunopathological reaction to the herpes virus, is the most likely pathophysiology. Combined immunosuppressive therapy was effective. Third, extensive arterial occlusions and PuR with macular ischemia made the visual prognosis limited. All three possibilities are relatively rare, with limited information in the extant literature.

The most relevant literature includes limited case reports and case series. Lee et al. (7) conducted 4 case series and an extensive literature review of 236 cases in which 105 cases (43.8%) were classified as idiopathic etiology. More bilateral manifestations were associated with younger age (<10 years) and better visual prognosis (7). A review by Walker et al. (1) of 57 case reports within 27 years (1976–2003) worldwide reported similar results in that nearly half of the cases were from the pediatric-age group. Most patients were characterized by Asian ethnicity and idiopathic etiology (1), including our case. The clinical presentation in the current case also coincides with another uncommon factor, non-necrotizing herpetic retinopathy, as reported by Bodaghi et al. (8) and Wensing et al. (9). The hallmark of the final diagnosis of the case was the absence of typical rapidly progressive necrotizing retinitis seen in acute retinal necrosis. As Bodaghi et al. (8) proposed, the constellation of papillitis and retinal vasculitis is an immunopathological phenomenon rather than a direct viral cytopathic effect. Therefore, systemic corticosteroids and immunosuppressive therapies were the mainstay of treatment with adjunctive low-dose prophylactic anti-viral agents in the current case.

The visual prognosis of FBA is excellent. However, similar to our case, a minority (10%) may present with poor final visual acuity (<0.1) due to structural complications such as macular pathologies, optic atrophy, and retinal vascular occlusions (1). Kwon et al. (10) reported a 39-year-old male with an unusual case of unilateral FBA associated with Behçet’s disease. Neovascularization of the disc was found, despite panretinal photocoagulation for non-perfusion areas. Foveal atrophy and disruption of the photoreceptor layer in the macular area developed with final vision limited to hand movement, 8 months later (10). In our patient, although initial macular edema responded favorably to treatment, macular ischemia with PuR was refractory to combined anti-inflammatory and antiplatelet therapy. Follow-up fluorescein angiography revealed extensive arterial and capillary dropout, and further neovascular complications, such as vitreous hemorrhage, retinal vascular occlusion, iris rubeosis, and neovascular glaucoma require close monitoring (7). As most ophthalmological treatment modalities, such as intravitreal anti-VEGF injections and panretinal photocoagulation, are only capable of suppressing VEGF release and avoiding further neovascular complications, few options are available to rescue retinal perfusion in such challenging scenarios. Therefore, HBOT is a viable option for physicians. As the patient had received numerous medications, it was not possible to evaluate the sole effect of HBOT. However, considering the significant structural changes in macular ischemia and foveal thinning on follow-up images (Figures 1C–F, 2D–H), the salvage effect of HBOT may have played a role in the visual recovery process.

Hyperbaric oxygen therapy is a treatment option for hypoxic tissue that increases tissue oxygen tension. It improves the oxygen supply because dissolved oxygen can diffuse into hypoxic tissue via tissue fluid, even if tissue vascularity is devastated. Most importantly, according to Henry’s law, the amount of dissolved oxygen increases in proportion to the increased partial pressure of oxygen. For instance, if 100% oxygen is breathed at 3 ATA (≈ 2,280 mmHg), dissolved oxygen rises from 0.31 to 6.02 vol%, which theoretically provides sufficient oxygen to maintain the basic metabolism of the human body without oxygen from hemoglobin (6). In an earlier animal study by Landers, the visual evoked response (VER) was restored to normal despite retinal artery occlusion while 1 ATA oxygen was administered. Normal VER indicated that the inner retinal layers were adequately oxygenated in this model (6, 11).

The human retina has a dual blood supply system (12). The retinal circulation supplies the inner layers of the retina (ganglion, bipolar, and Muller glial cells) and the choroidal circulation supplies the outer layers (photoreceptors and retinal pigment epithelium) (12). Therefore, in the model of central retinal artery occlusion, it is postulated that higher partial pressure of oxygen could diffuse farther from the choroidal circulation or other patent retinal vessels to reach the ischemic retina using HBOT (13). HBOT should be able to lessen the degree of ischemia neuronal injury and restart cellular metabolism. The circumstance of ischemic neuronal damage within the retina begins with a hypoxia event, just as it takes place in the ischemic stroke within central nervous system (14). According to Kim et al., patients with central retinal artery occlusion (CRAO) benefit from HBOT, with greater visual improvement (5). HBOT is not only supposed to improve visual acuity via increased oxygen concentration to ischemic retinas, it also reduces retinal apoptosis according to animal models (4, 15). Recently, another case demonstrated visual acuity improvement for mumps-associated FBA after sessions of HBOT (16).

The pathophysiology of PuR remains uncertain, but the most widely accepted theory is an embolic phenomenon, resulting in occlusion of the precapillary arterioles and subsequently ischemia (3). We believed that HBOT could also improve tissue oxygenation to the macular ischemia. Lin et al. reported HBOT improved visual function and retinal appearance in a case with Purtscher’s retinopathy secondary to chest injury (17). In addition, Haji and Frenkel also reported a case of radiation-induced macular ischemia, who benefited from HBOT with macular perfusion improvement (18). In the present case, signs of avascular area and vasculitis appeared at the first visit. Although HBOT was not initiated immediately after diagnosis, visual acuity steadily improved under sessions of HBOT with successful corticosteroid tapering.

The novel information provided by this case is that the prognosis of FBA is not always favorable. With concurrent structural complications, such as macular pathologies, optic atrophy, and retinal vascular occlusions, aggressive corticosteroid with combined immunomodulatory therapy is necessary. We recommend early intervention with HBOT to salvage severe macular ischemia. Long-term management should monitor for and attempt to prevent neovascular complications.

## Conclusion

Hyperbaric oxygen therapy may be a beneficial rescue treatment for retinal ischemia secondary to FBA with PuR. Further clinical and basic research is needed to evaluate the effectiveness of HBOT for uveitis with occlusive retinal vasculitis.

## Ethics statement

The study was approved by the FEMH Ethics Committee in Taiwan (FEMH-111106-C). Written informed consent for publication was obtained from the involved patient and his parents. Written informed consent to participate in this study was provided by the participants’ legal guardian/next of kin.

## Author contributions

C-TL and H-TC: conceptualization. T-HH: data curation. H-TC: funding acquisition and supervision. T-HH and ZZ: investigation. Y-RH: methodology and resources. C-CC and J-HW: project administration. C-TL, T-HH, and ZZ: writing—original draft. Y-RH, H-TC, and J-KW: writing—review and editing. All authors contributed to the article and approved the submitted version.
